# HPV-Induced MiR-21 Promotes Epithelial Mesenchymal Transformation and Tumor Progression in Cervical Cancer Cells through the TGF*β* R2/hTERC Pathway

**DOI:** 10.1155/2022/6297694

**Published:** 2022-09-01

**Authors:** Ying Han, Qiuhong Li, Chenqi Ling, Ming Jin, Dongdong Li, Jie Zhong, Li Wang

**Affiliations:** Department of Gynecology, Yangpu District Shidong Hospital Affiliated to Shanghai University of Technology, Shanghai 200438, China

## Abstract

Cervical cancer (CC) is a common malignant tumor in women. It ranks first among the malignant tumors of woman reproductive organs and is one of the most important cancers in the world. Current studies suggest that human papillomavirus (HPV) infection, especially high-risk persistent infection, is the basic cause of cervical precancerous lesions and cervical cancer. MicroRNA-21 (miR-21) plays a role similar to oncogenes in the occurrence and growth of malignant tumors and can be developed as a potential target for treating malignant tumors. Recently, the study of the mechanism of malignant invasion and metastasis has made great progress. The current consensus is that the invasion and metastasis of malignant tumors is a complicated biological process with multistep and multigene control; the process of epithelial mesenchymal transition (EMT) may be the initial event of invasion and metastasis of epithelial malignant tumors. EMT means that epithelial cells obtain the characteristics of mesenchymal cells, which has main characteristics such as the loss of epithelial cell characteristics and the achievement of mesenchymal cell features, and then induce epithelial cells to acquire the ability of migration and invasion, and participate in many physiological and pathological processes of human body, including embryogenesis, organ differentiation, tissue inflammation, and wound healing. Research has proved that miR-21 is associated with the invasion and metastasis of cervical cancer, and its specific mechanism has not been completely clear; EMT exerts a significant effect on the invasion and metastasis of epithelial malignant tumors; we speculate whether miR-21 regulates the EMT process of cervical cancer cells. ELISA and RT-PCR studied HPV-induced cervical cancer cells, and it was found that HPV may induce miR-21 to pass through the TGF *β* R2/hTERC pathway which promotes epithelial stromal transformation and tumor progression of cervical cancer cells.

## 1. Introduction

The incidence of cervical cancer is the second most common malignancy of the female reproductive system, second only to breast cancer. There are above 500,000 new cases worldwide every year, most of which are in developing countries [1–3]. China is a big country with above 130,000 new cases of cervical cancer every year, and more than 60,000 deaths due to cervical cancer every year [4, 5]. Recently, with the use of HPV vaccine, cervical cancer screening methods include early screening, secondary prevention, and other methods, and its incidence rate has decreased, but because the HPV vaccine is still not in the world within the scope of application, comprehensive economic underdeveloped regions are still in early screening; cervical cancer death rates remain high, and is still one of the diseases which cause serious damage to the health of women [6, 7]. As is known to all, invasion and metastasis are the major reasons for poor prognosis of cervical cancer. Therefore, a detailed and systematic study on the molecular mechanism of invasion and metastasis is of great significance to carry out individualized targeted intervention and treatment.

The relationship between microRNAs and tumors has always been a hot theme in the field of tumor research recently. MicroRNAs are a class of endogenous noncoding single-stranded RNA molecules with a length of about 18–25 nt [8–10]. They control gene expression at the posttranscriptional level by complementary binding with the 3′ noncoding region (3′-UTR) of the target mRNA, leading to mRNA degradation or translation inhibition, and participate in a series of important life processes, including cell proliferation, differentiation malignant transformation, and apoptosis. Mierornas regulate about one third of human gene expression, and are closely associated with the occurrence, growth, invasion and metastasis of malignant tumors [11–13]. Among them, microRNA-21 (miR-21) is a kind of microRNA discovered earlier and studied more. It is highly expressed in various malignant tumor tissues and cells. Through acting on a variety of tumor suppressors, such as PDCD4, PTEN, Maspin, BMPRII, and Sprouty2, the dysregulated miR-21 participates in the proliferation, invasion, metastasis, antiapoptosis, and other biological behaviors of malignant tumor cells; miR-21 plays a role similar to oncogenes in the occurrence and growth of malignant tumors, and can be developed as a potential target for the treatment of malignant tumors. A lot of research have shown that the expression of miR-21 is elevated in cervical cancer. At present, it is known that the continuous infection of high-risk human papillomavirus (HPV) is the major cause of cervical cancer [14]. After HPV is integrated into the host cell genome, it can lead to a change in integrated cytogenetics and lead to its cancer. The human miR-21 gene is located in fral7b, the fragile site of chromosome 17q23.2, which happens to be the site where HPVl6 is easy to integrate. It can be speculated that the miR-21 gene adjacent to the HPV integration site may be related to its increased expression level in cervical cancer. It was also found that the proliferation of HeLa cells was significantly inhibited after inhibiting the expression of miR-21 in the HeLa cell line of cervical cancer. It was observed that miR-21 could regulate the proliferation, apoptosis, invasion, and metastasis of cervical squamous cell carcinoma cells by controlling the expression of its target gene CCL20. In addition, the expression of miR-21 in cervical cancer is related to the clinical stage and lymphatic metastasis of cervical cancer patients. These studies fully show that miR-21 is closely associated with the occurrence and growth of cervical cancer, but the specific molecular mechanism of miR-21 regulating the invasion and metastasis of cervical cancer has not been fully understood [15, 16].

Recently, the study of the mechanism of malignant invasion and metastasis have made great progress. The current consensus is that the invasion and metastasis of malignant tumors are a complicated biological process with multistep and multigene control, including local infiltration of tumor cells, penetration into the blood vessel wall, transport, penetration out of the blood vessel wall, and distant planting. The process of epithelial mesenchymal transition (EMT) may be the initial event of invasion and metastasis of epithelial malignant tumors. EMT means that epithelial cells obtain the characteristics of mesenchymal cells, which has main characteristics such as the loss of epithelial cell characteristics and the achievement of mesenchymal cell features, and then induce epithelial cells to acquire the ability of migration and invasion, and participate in many physiological and pathological processes of human body, including embryogenesis, organ differentiation, tissue inflammation, and wound healing [16, 17]. EMT is characterized by cell metastasis and invasion, which of course includes the invasion and metastasis of tumor cells. Previous research has confirmed that EMT exerts a key effect on the primary invasion and secondary metastasis of various epithelial malignant tumors. It has been found that various signaling pathways take part in the EMT process of tumors, among which the transforming growth factor-*β* (TGF-*β*) exerts a significant effect. Research has proved that miR-21 is associated with the invasion and metastasis of cervical cancer, and its specific mechanism has not been completely clear. EMT exerts a significant effect on the invasion and metastasis of epithelial malignant tumors [18–21]. We speculate whether miR-21 can drive the invasion and metastasis of cervical cancer cells by regulating the EMT process of cervical cancer cells. At present, there is no relevant report at home and abroad.

This research aimed to explore the association between miR-21 and invasion and metastasis of cervical cancer, the relationship between key molecules of EMT process and invasion and metastasis of cervical cancer, and the relationship between miR-21 and key molecules of EMT process. In vitro cell experiments were conducted to further verify the effect of miR-21 on the EMT process, invasion, and metastasis of cervical cancer cells, and to reveal whether miR-21 affects the invasion and metastasis of cervical cancer cells by regulating the EMT process, to provide experimental data and theoretical basis for finding relevant targets of cervical cancer invasion and metastasis, stopping the invasion and metastasis process of cervical cancer, and carrying out gene-targeted intervention and individualized treatment.

## 2. Methods

### 2.1. Cells

Three kinds of human cervical cancer cell lines: HPV18 (+) Hela (CL-0101), HPV16 (+) Siha (CL-0048 CL-0210), and HPV (−) C33A (CL-0045) (offered by the Cell Bank of The Committee for Typical Culture Preservation of Chinese Academy of Sciences).

### 2.2. Cell Resuscitation, Culture, Passage, and Freezing

Siha cell line was HPV type 16 (HPV16+) cervical squamous cell line, Hela cell line was HPV type 18 (HPV18+) cervical squamous cell line, and C33a was HPV negative (HPV−) cervical squamous cell line. For cell recovery, the principle of fast melting was observed. First, the water bath was adjusted to 37°C, and the frozen storage tube was taken out from the liquid nitrogen tank and quickly put into the 37°C water bath for rapid melting. Then, the cell suspension was sucked out with a pipette, injected into the centrifugal tube and added with 4 mL complete culture medium, centrifuged at 1000 r/min for 5 min, and the supernatant was discarded. A proper amount of culture liquid was added to blow and make it form suspension. Siha cells, Hela cells, and C33a cells were cultured under the same conditions: The fine culture was carried out in a DMEM medium containing 10% high-quality fetal bovine serum and 1% penicillin-streptomycin double antibody. The medium was changed once from 24 to 48 h, and the culture was carried out at 37°C in 5% carbon dioxide and CO_2_ saturated humidity. When the degree of cell fusion reached about 90%, the operation was carried out on the ultra-clean workbench, the old medium was discarded and washed with PBS 3 times. Trypsin digestion solution was added into the 25 cm culture flask for about 0.5–1.0 ml and placed in the incubator at 37°C for about 1.5 min. The bottom of the flask was gently vibrated to make all the cells shed, and 3 mL of complete medium was added. The cell suspension was gently blown, and the supernatant was collected in the centrifuge tube and discarded. Then, the complete culture medium was added and the cell suspension was blown, and the culture flask was placed in a 37°C incubator at a ratio of 1 : 2. The principle of slow freezing should be followed when cells are cryopreserved, and cells growing at logarithmic stages should be selected, preferably after 4 or 5 generations of subculture. The culture medium was centrifuged and the supernatant was removed and left for cell precipitation, the cryopreservation solution was added(10% DMSO + 90% FBS), blown and mixed well, and put into cell a cryopreservation tube by 1 mL per tube.

### 2.3. ELISA

Cells were collected from the 6-well plate, cell lysis solution was added, and the extracted proteins were quantified by the BCA protein quantification kit and stored separately (−80°C). The levels of TGF*β* R2 and hTERC were detected by kit method.

### 2.4. RT-PCR Assay

1 ml of trizol was added to the 6-well plate to lyse the cells and was placed for 5 min, 0.2 ml of chloroform was added and mixed well and left to stand at room temperature for 3 min. The mixture was centrifuged at 10 000 r/min for 10 min. The supernatant was taken and an equal volume of isopropanol was added, it was left to stand for 10 min. The mixture was again centrifuged at 10 000 r/min for 10 min. The supernatant was discarded and 1 ml of 75% ethanol/tube was added. It was centrifuged at 7500 r/min for 5 min. the supernatant was discarded and the sediment was dissolved with an appropriate amount of DEPC water. The concentration and purity of RNA were measured by an ultraviolet spectrophotometer (Nano drop 1000). The mRNA expressions of miR-21, TGF *β*R2, and hTERC were detected.

### 2.5. Statistical Analysis

SPSS 20.0 statistical software was adopted for data analysis, and the measurement data was shown as mean ± standard deviation (*x* ± *s*). One way variance homogeneity test was conducted first when comparing the two groups, and Tukey HSD method was used and Tukey HSD method was used for homogeneity of variance; when the variance is uneven, the rank sum test of two independent samples in the nonparametric test is used. *P* < 0.05 was statistically significant.

## 3. Results

### 3.1. HPV Induced Increased Levels of TGF *β* R2

Compared with the HPV (−) uterine cervical carcinoma cell C33A, the contents of TGF *β* R2 in HPV16 (+) Siha and HPV18 (+) Hela were greatly increased in Table 1 (*P* < 0.05).

### 3.2. HPV Induced Increased Expression of miR-21

Compared with the HPV (−) uterine cervical carcinoma cell C33A, the expression of miR-21 in HPV16 (+) Siha and HPV18 (+) Hela were greatly increased in Figure 1 (*P* < 0.05).

### 3.3. HPV Induced Increased Expression of TGF β R2

Compared with the HPV (−) uterine cervical carcinoma cell C33A, the expression of TGF *β* R2 in HPV16 (+) Siha and HPV18 (+) Hela were significantly increased in Figure 2 (*P* < 0.05).

### 3.4. HPV Induced Increased Expression of hTERC

Compared with the HPV (−) uterine cervical carcinoma cell C33A, the expression of hTERC in HPV16 (+) Siha and HPV18 (+) Hela were greatly increased in Figure 3 (*P* < 0.05).

## 4. Discussion

Cervical cancer is one of the most common malignant tumors endangering women's health, accounting for the fourth place in the total number of female cancer deaths in the world, 85% of which come from developing countries. Currently, it is known that the major cause of cervical cancer is the continuous infection of high-risk HPV virus [22]. Although the overall incidence rate of cervical cancer has decreased with the development of primary and secondary cancer prevention measures such as HPV vaccine application and cervical cancer early screening technology, due to the imbalance of global economic development, the incidence rate has not decreased significantly in developing countries, and the mortality is still high. China is a large country of cervical cancer, with nearly 130000 new cases each year, accounting for one third of the global number of cervical cancer [23–26]. There are as many as 60000 deaths due to cervical cancer every year. Recently, the incidence of cervical cancer is still young. Cervical cancer has become an important disease seriously endangering the health of Chinese women [27]. Hence, it is especially significant to study the mechanism of the occurrence and growth of cervical cancer, including HPV infection, cervical intraepithelial neoplasia, cervical carcinoma in situ, and early invasive cancer. The occurrence and growth of invasive carcinoma to distant metastasis is a continuous process, which must involve the abnormal expression of a variety of coding genes and noncoding genes [28]. Any process can become the target of blocking intervention. It is known that the main cause of poor prognosis of cervical cancer is local invasion and distant metastasis. Preventing invasion and metastasis is the key to improve the prognosis [29]. Therefore, a detailed and systematic study on the molecular mechanism of invasion and metastasis of cervical cancer is greatly significant for individualized targeted intervention and treatment.

Since 1993, microRNAs have been hot in the field of tumor study. MicroRNAs regulate gene expression mainly by binding to the 3′-UTR base of target mRNA, inhibiting mRNA translation or directly degrading it, and play a significant effect on the pathogenesis and progress of malignant tumors. MicroRNAs influence the proliferation, invasion, metastasis, and apoptosis of tumor cells by controlling the expression of tumor suppressor genes or oncogenes, or directly as tumor suppressor genes or oncogenes [7–10]. With the development of gene chip, real-time quantitative PCR, Northern blot and other molecular biological technologies, and more and more microRNAs related to malignant tumors have been found. MiR-21, a kind of microRNA discovered earlier, studied more, and paid more attention, is also closely related to malignant tumors [30–32]. The abnormal expression of miR-21 and its important role in the occurrence and growth of these malignant tumors have been confirmed in the relevant studies of glioma, gastric cancer, colon cancer, liver cancer, lung cancer, breast cancer, cervical cancer, and other tumors. This research found that miR-21 of HPV-induced cervical cancer cells was significantly increased by RT-PCR.

Epithelial mesenchymal transition (EMT) is a dynamic process in which polar epithelial cells are transformed into mesenchymal cell phenotypes through complex biochemical changes, which enhances the ability of infiltration and metastasis, improves the tolerance to apoptosis, and largely changes the composition of extracellular matrix. However, in some cases, this process can be reversed, that is, mesenchymal epithelial transformation (MET) [33]. It has been found that epithelial cells promote the formation of embryos and organs through the transformation of EMT and MET. In addition, EMT can also be activated in various inflammation and tumors. Now, it is generally accepted that the process of EMT is the formation mechanism of stromal cells during cell formation and tissue damage during embryonic differentiation, and leads to the infiltration and metastasis of tumor cells in epithelial tumors. In this process, epithelial markers including cadherin decreased or lost, and interstitial markers such as wavy protein and fibronectin increased. It was found that silencing HPVl6 E7 in human skin keratinocytes could increase the expression of cadherin, an epithelial marker. Consistent with this, in this experiment, after the E6 and E7 genes of HPVl6 and HPVl8 viruses were silenced, respectively, the expression of cadherin and the marker of EMT increased, while the expression of N-cadherin and b-catenin decreased; that is, the process of mesenchymal epithelial transformation occurred, the degree of tight junction between cells increased, and the ability of migration decreased, that is, the capacity of tumor cells to invade, infiltrate, and metastasize decreased [34, 35]. In other words, the E6 and E7 genes of HPV16 and HPV18 may promote the malignant progression of cervical epithelial cells by promoting the process of epithelial stromal transformation. Among the many signal pathways that mediate EMT in tumor cells, the TGF *β* signal pathway is an important member. TGF *β* is an important subclass of TGF. It is a multifunctional polypeptide molecule, which can regulate cell proliferation, differentiation, embryonic development, and wound repair. Studies have observed that the high expression of TGF *β* is associated with many tumor kinds including breast cancer, prostate cancer, liver cancer, lung cancer, and colon cancer. In tumor tissues including cervical cancer, high levels of TGF-*β*1 often represent the type with higher invasiveness, which indicates that patients' prognosis is poor, and many tumor cells' positive response to TGF-*β*1 represents higher invasiveness. TGF *β* can mediate the process of EMT in tumor cells and nontumor epithelial cells, and studies have confirmed that TGF-b1 promotes the process of epithelial mesenchymal transformation in SiHa cells. Some research has also shown that the high expression of TGF *β* is closely associated with the progression of CIN to cancer through the study of exfoliated cells in Pap smear. In addition, HPVl6 E6 and E7 genes enhanced the activity of TGF *β* promoter. Our study further confirmed and extended these views, HPV induced increased TGF *β*R2 expression [34, 35].

It is found that human telomerase consists of human telomerase reverse transcriptase (hTERT), human telomerase RNA component (hTERC), and pseudouracil synthase. The researchers used a variety of methods to find the expression of hTERC gene in normal cervical tissues, cervical CIN lesions, and cervical cancer. The outcomes displayed that hTERC was positive in cervical cancer group, and its activity was significantly higher than the other two groups. The results of this experiment were the same. Therefore, the activity of hTERC is expected to become a tumor marker [9]. Studies have shown that high-risk HPV infection can lead to the amplification of TERC gene, and HPV infection, as an initiating factor, can lead to the reactivation of telomerase gene, both of which trigger cell proliferation [10]. The results showed that HPV could induce the increase of hTERT expression. Therefore, we speculate that HPV may induce miR-21 to pass through the TGF *β* R2/hTERC pathway which promotes epithelial stromal transformation and tumor progression of cervical cancer cells.

The significance of cell function test is not only here, but also in treating cervical cancer. Currently, the treatment of cervical cancer is mostly radical surgery and radiotherapy, and surgical trauma and the toxic and side effects of radiotherapy will greatly reduce the quality of life of patients. Since miR-21 exerts a main effect on driving the occurrence and growth of cervical cancer, we found that no matter cervical squamous cell carcinoma or adenocarcinoma cell lines, the expression of miR-21 in cells is inhibited, and the invasion and metastasis ability of cells is inhibited, which offers a new idea for treating cervical cancer, suggesting that miR-21 can become a target for the treatment of cervical cancer. By interfering with the expression of miR-21, it can block the occurrence, growth, invasion, and metastasis of cervical cancer. The research on the target genes that confirm the direct role of miR-21 in EMT of cervical cancer needs to be further implemented in the future. In addition, further tumor formation experiments in animals need to be carried out to improve the regulation theory of miR-21 on EMT process and invasion and metastasis process of cervical cancer cells.

## 5. Conclusion

In conclusion, miR-21 of HPVl6 and HPVl8 may pass through during the progression of cervical cancer and the TGF *β*R2/hTERC signaling pathway mediates the process of epithelial mesenchymal transformation, thereby enhancing the ability of tumor cells to proliferate, infiltrate, and metastasize. However, whether it can be affected by other ways and other factors needs further research, which may offer a new goal for treating cervical cancer.

## Figures and Tables

**Figure 1:** HPV induced increased expression of miR-21.

**Figure 2:** HPV induced increased expression of TGF *β* R2.

**Figure 3:** HPV induced increased expression of hTERC.

**Table 1:** The levels of TGF *β* R2 and hTERC by ELISA were detected.

	HPV (−) C33A	HPV16 (+) Siha	HPV18 (+) Hela
TGF *β* R2	13.25 ± 1.42	18.74 ± 2.02^*∗*^	20.19 ± 2.17^*∗*^

## Data Availability

The datasets used and analyzed during the current study are available from the corresponding author upon reasonable request.
